# Thyrocyte-specific inactivation of *p53* and *Pten* results in anaplastic thyroid carcinomas faithfully recapitulating human tumors

**DOI:** 10.18632/oncotarget.380

**Published:** 2011-12-20

**Authors:** Valeria G. Antico Arciuch, Marika A. Russo, Mariavittoria Dima, Kristy S. Kang, Florence Dasrath, Xiao-Hui Liao, Samuel Refetoff, Cristina Montagna, Antonio Di Cristofano

**Affiliations:** ^1^ Department of Developmental and Molecular Biology, Albert Einstein College of Medicine, Bronx, NY; ^2^ Department of Genetics, Albert Einstein College of Medicine, Bronx, NY; ^3^ Department of Medicine, University of Chicago, Chicago, IL; ^4^ Department of Pediatrics and Committee on Genetics, University of Chicago, Chicago, IL

**Keywords:** thyroid cancer, mouse model, anaplastic, glycolysis, PI3K, Pten, p53

## Abstract

Anaplastic thyroid carcinoma (ATC) is the most aggressive form of thyroid cancer, and often derives from pre-existing well-differentiated tumors. Despite a relatively low prevalence, it accounts for a disproportionate number of thyroid cancer-related deaths, due to its resistance to any therapeutic approach. Here we describe the first mouse model of ATC, obtained by combining in the mouse thyroid follicular cells two molecular hallmarks of human ATC: activation of PI3K (via *Pten* deletion) and inactivation of *p53*. By 9 months of age, over 75% of the compound mutant mice develop aggressive, undifferentiated thyroid tumors that evolve from pre-existing follicular hyperplasia and carcinoma. These tumors display all the features of their human counterpart, including pleomorphism, epithelial-mesenchymal transition, aneuploidy, local invasion, and distant metastases. Expression profiling of the murine ATCs reveals a significant overlap with genes found deregulated in human ATC, including genes involved in mitosis control. Furthermore, similar to the human tumors, [*Pten, p53*]^thyr−/−^ tumors and cells are highly glycolytic and remarkably sensitive to glycolysis inhibitors, which synergize with standard chemotherapy. Taken together, our results show that combined PI3K activation and p53 loss faithfully reproduce the development of thyroid anaplastic carcinomas, and provide a compelling rationale for targeting glycolysis to increase chemotherapy response in ATC patients.

## INTRODUCTION

Thyroid cancer is the most common endocrine neoplasm, and one of the few tumor types for which incidence has been increasing over the past 20 years [1]. Well-differentiated thyroid cancers (papillary and follicular) have generally a good prognosis and can be effectively managed through a combination of surgery and radioactive iodine treatment [2]. Anaplastic thyroid carcinoma (ATC) represents the most aggressive and undifferentiated subtype of thyroid cancer. It often coexists with well-differentiated tumors, suggesting that it arises from pre-existing follicular or papillary tumors [3, 4]. Although it comprises less than 5% of thyroid malignancies, ATC accounts for up to 40% of deaths from thyroid cancer [5]. In fact, ATC is almost invariably lethal, with no effective therapy available [6, 7]. Thus, its median survival of around 4 months, due to rapid onset, tracheal and esophageal invasion, and uncontrolled metastases to the lungs and, to a less extent, to bones, skin and brain, has not changed in more than half a century [8]. Dedifferentiation, a hallmark of ATC, is manifested by loss of specific thyroid cell characteristics and functions, including expression of thyroglobulin, thyroid peroxidase, thyroid stimulating hormone receptor and the Na/I symporter, NIS [9]. Other ATC characteristics include pleomorphism, with often coexisting areas of squamoid, spindle cell, and giant cell morphology [10], epithelial-to-mesenchymal transition [7], and neutrophilic infiltrate [11].

Molecular characterization of ATCs has revealed a high degree of chromosomal instability and aneuploidy [12]. In addition, common alterations in a number of signal transduction pathways have been identified. Molecular changes that characterize ATC have been recently reviewed in a number of publications [9, 13, 14], and involve most often *p53* loss or inactivation, and activation of the PI3K cascade, of RAS family members, or of BRAF.

One major obstacle to the development of more effective therapeutic approaches to ATC has been the lack of an immunocompetent, autochthonous mouse model closely recapitulating the clinicopathological features of human ATC. In spite of significant advancements, most genetically engineered mouse models described to date only develop differentiated thyroid cancer, such as PTC [15-17] and FTC [18-20]. One notable exception is represented by the *Braf*^V600E^ transgenic model, which develops poorly differentiated foci from concurrent papillary lesions [21]

In this study, we report the characterization of the first mouse model of ATC, based on the simultaneous activation of the PI3K signaling cascade and inactivation of *p53* in the mouse thyroid epithelial cells. The tumors developing in these mice closely phenocopy human ATCs, undergo the glycolytic shift known as Warburg effect, and are highly sensitive to the therapeutic use of glycolytic inhibitors. Thus, this model represents a novel, powerful tool to understand the biology of human thyroid anaplastic carcinomas, and to develop innovative therapeutic approaches for what is today still a lethal disease.

## RESULTS

### Anaplastic thyroid carcinoma development in [*Pten, p53*]^thyr−/−^ mice

Mice with a targeted deletion of the *Pten* tumor suppressor gene in the thyroid follicular cells exhibit constitutive PI3K pathway activation and develop, from birth, hyperplastic glands that progress to nodular lesions by 6-10 months of age [22] and to well-differentiated follicular carcinomas after one year of age [19]. Building on available clinicopathological data that point at *p53* as the most commonly mutated or deleted gene in anaplastic thyroid tumors, we crossed the *Pten* mutants with mice carrying a floxed *p53* allele in order to model more aggressive thyroid tumors. Thyroid-specific *p53* loss did not cause any overt phenotype (Figure 1A and data not shown). Conversely, concomitant loss of p53 dramatically reduced the survival of *Pten*^thyr−/−^ mice (median survival 38.4 weeks vs. 75.3 weeks), while reduction to heterozygosity of either allele, in the absence of the other, resulted in an intermediate phenotype (median survival: 61.3 weeks for [*Pten*^thyr−/−^, *p53*^thyr+/−^] mice, and 58.45 weeks for [*Pten*^thyr+/−^, *p53*^thyr−/−^] mice) (Figure 1A). Similar to *Pten*^thyr−/−^ mice, [*Pten, p53*]^thyr−/−^ compound mutants displayed drastically reduced Thyroid-Stimulating Hormone (TSH) serum levels. However, the absence of significantly increased T4 hormone levels suggests that TSH suppression is not the consequence of relieving the physiological negative feedback normally induced by elevated thyroid hormone levels (Figure 1B, C).

**Figure 1:** Clinicopathological features of [*Pten, p53*]^thyr−/−^ mice (A) Kaplan-Meyer analysis of the effect of progressive *p53* deletion on the survival of *Pten*^thyr−/−^ mice. (B, C) TSH and T4 serum levels in control, single mutant and double mutant (DM) mice. (D-K) Histopatological features of tumors developing in [*Pten, p53*]^thyr−/−^ mice. (D) Anaplastic carcinoma (left) flanking an area of well-differentiated follicular carcinoma (right). Undifferentiated tumors display areas of spindle cell morphology (E), with frequent giant cells (F), and occasional bone metaplasia (G). Tumors invade locally into the muscle (H), and the trachea (I), and metastasize to the lungs (J) or, sporadically, to the liver (K). Bar: 100μm.

Post mortem analysis of 8-10 month old [*Pten, p53*]^thyr−/−^ mutants revealed in all cases a strikingly enlarged thyroid gland (average gland weight 392±350 mg, vs. 3.7±1.1 mg in age-matched controls) causing severe tracheal compression and adhering to adjacent tissues. Histopathological analysis showed the coexistence of small remnants of well-differentiated follicular carcinomas, similar to those developing in aging *Pten*^thyr−/−^ mice, and of more extensive pleomorphic areas (Figure 1D) exhibiting, as in human anaplastic carcinomas, spindle cell morphology (Figure 1E), giant, osteoclast-like, multinucleated cells (Figure 1F), and even areas of osseous metaplasia (Figure 1G). These aggressive tumors invaded locally into the muscle (Figure 1H) and trachea (Figure 1I) and, in 28% of mice, metastasized to the lungs (Figure 1J) or, albeit less often, to the liver (Figure 1K). Conversely, analysis of thyroids from 4-8 month old [*Pten, p53*]^thyr−/−^ mice only showed areas of well differentiated follicular carcinomas, indistinguishable from those developing in older *Pten*^thyr−/−^ mice (data not shown). Thus, combined loss of *p53* and PI3K activation in the thyroid follicular cells results in the development of aggressive, metastatic tumors closely resembling human thyroid anaplastic carcinomas.

### Mouse ATCs undergo dedifferentiation, genomic instability, and EMT

Loss of thyrocyte differentiation is a hallmark of human ATC. We used real time PCR to measure the expression levels of a panel of genes associated with thyroid differentiation and function in freshly dissected glands and tumors. Expression of the *Foxe1*, *Pax8*, and *Nkx2-1* transcription factors, as well as of the thyroid-specific genes *Duox2*, *Tpo*, *Tg*, *Tshr*, and *Slc5a5* (*Nis*) was generally not altered in single mutants nor in [*Pten, p53*]^thyr−/−^ mice up to 8 months of age, before the development of frank ATC. However, expression of each of these markers was reduced to almost undetectable levels in every anaplastic tumor analyzed (Figure 2), supporting the notion that the tumors developing in the compound mutants are indeed undifferentiated carcinomas.

**Figure 2:** Expression profiling by real-time PCR of a panel of thyroid differentiation markers using thyroid pools from 4-month old control and single mutant mice, ATC-free, progressively older (4, 6, 8 months) double mutants, and histologically confirmed ATCs from 8- to 9-month old double mutants.

A second frequent aspect of human ATC is an elevated degree of genomic instability, leading to marked aneuploidy. We analyzed metaphase spreads from early passage primary cultures of several histologically confirmed anaplastic carcinomas, and found that these cells were invariably aneuploid (Figure 3A), with evidence of widespread chromosomal damage, including chromosome and chromatid breaks, complex rearrangements, translocations, premature centromere division, and the presence of chromosomal debris (Figure 3B). Thus, combined loss of the *Pten* and *p53* tumor suppressors leads to tumors that display genomic instability.

**Figure 3:** Mouse ATCs display chromosomal instability and aneuploidy (A) Chromosome counts in two representative early passage (p2) primary cultures from histologically confirmed ATCs. Note the wide distribution of chromosome numbers within the same culture. (B) Karyotypic analysis of two representative cells from independent tumors, showing chromatid breaks (thick arrows), chromosome breaks (thin arrows), translocations (#), and complex rearrangements (*).

To further validate the [*Pten, p53*]^thyr−/−^ strain as a model of human ATC, we performed immunohistochemistry on paraffin sections from 9-10 month old mice displaying both well-differentiated and undifferentiated tumor areas in order to determine whether these tumors display epithelial-to-mesenchymal transition (EMT). Strikingly, the undifferentiated area of all the tumors analyzed had lost the expression of the epithelial marker E-cadherin, had acquired the expression of the mesenchymal marker Vimentin, and displayed high levels of phosphorylated Smad2 (Figure 4). No EMT was detected on thyroid sections from younger mice (not shown). These data show that the tumors developing in the compound mutants invariably undergo EMT, and strongly suggest that this process is, at least in part, under the control of elevated Tgf-β signaling.

**Figure 4:** [*Pten, p53*]^thyr−/−^ ATCs undergo EMT (A) H&E staining of a representative tumor area containing both a follicular carcinoma (left) and an anaplastic carcinoma (right) component. (B-D) Immunohistochemical detection of phospho-Smad 2 (B), E-cadherin (C), and vimentin (D). Bar: 100μm.

A large subset of human ATCs is characterized by activating *BRAF* or *RAS* mutations. To determine whether the ATCs developing in [*Pten, p53*]^thyr−/−^ mice have somatic activating mutations in either *Braf* or in one of the three *Ras* genes, we sequenced the known hotspots (*Braf* exons 11 and 15, H-; N-, and *Kras* exons 1 and 2) in five cell lines established from tumors developed by [*Pten, p53*]^thyr−/−^ double mutant mice. All cell lines had wild type sequences, strongly suggesting that neither *Braf* nor *Ras* isoforms are involved in ATC development in this mouse model (data not shown).

### ATCs are addicted to driver gene signaling

Loss of *Pten* is anticipated to lead to constitutive phosphorylation of Akt and deregulation of its downstream targets. Indeed, western blot analysis of thyroid extracts from control, single, and young double mutants showed elevated pSer^473^-Akt, pThr^389^-S6k, and pSer^240/244^-S6 in thyroids lacking *Pten* (Figure 5A). Double mutant glands also displayed moderate levels of pERK1/2. ATCs were characterized by a somewhat increased phosphorylation of S6, and by variable levels of pERK1/2. However, when phosphorylation and activation of these proteins was examined by IHC, we found that Akt phosphorylation was higher in the remnants of well-differentiated lesions within the tumor than in the anaplastic component, which instead showed higher levels of pS6 (Figure 5B). This finding suggests that the well-known negative feedback mediated by S6k and IRS-1 [23] might be favored or enhanced in ATCs. Furthermore, it may underline a reduced dependence of fully developed ATCs on Akt signaling.

**Figure 5:** ATCs are addicted to driver gene signaling (A) Western blotting analysis of the activation status of Akt and MAPK pathways in 4-month old control and single mutant mice, ATC-free, progressively older (4, 6, 8 months) double mutants, and histologically confirmed ATCs from 8- to 9-month old double mutants. (B) immunohistochemical detection of activated Akt, S6 ribosomal protein, and ERK1/2 in tumor areas with both well-differentiated and anaplastic components. (C) IC_50_ values for an Akt inhibitor (MK-2206) and a MEK inhibitor (U0126) in a panel of mouse and human anaplastic (ATC) and follicular (FTC) carcinoma cell lines. On the bottom, a Western blotting showing the effect on the activation of Akt and ERK1/2 of one hour exposure to these inhibitors (MK-2206: 500nM, U0126: 10μM).

In the same tumors, ERK1/2 activation was restricted to scattered patches of cells, often near the invasive edges of the undifferentiated components.

The accumulating genetic alterations consequent the high degree of genomic instability within ATCs might alter the dependence of these tumors on their driver oncogenic alteration, i.e. increased Akt signaling. We used two cell lines, T1860 and T1903, which we have derived from anaplastic tumors developed by [*Pten, p53*]^thyr−/−^ mice, to determine the sensitivity of these murine ATCs cells to specific pathway inhibition, and compared them to the human follicular carcinoma line FTC-133 (*PTEN* and *p53* mutant), and the human ATC lines CAL-62 (*KRAS* and p53 mutant) and C643 (*HRAS* and p53 mutant). One-hour treatment with the AKT inhibitor MK-2206 (0.5μM) or with the MEK inhibitor U0126 (10μM) effectively abolished AKT and ERK1/2 phosphorylation in all cell lines (Figure 5C). The effect of both compounds on cell viability, measured by determining the IC_50_ after 72h treatment, clearly correlated with the cell lines' genetic makeup, with *Pten*^−/−^ cells being more sensitive to AKT inhibition than *Pten*^+/+^ cells, and *Ras* mutant cells more sensitive to MEK inhibition than cells with wild type *Ras* (Figure 5C).

Thus, although mouse ATCs display lower pAkt levels than coexisting well-differentiated tumor areas, they still depend on Akt signaling for their survival and proliferation.

### A “mitotic gene signature” in mouse and human ATCs

To gain insight into the molecular characteristics of ATCs developed by [*Pten, p53*]^thyr−/−^ mice, we performed genome-wide expression profiling using the Affymetrix platform on thyroids from 3-month old control, single, and double mutant mice, as well as on five follicular and five anaplastic carcinomas developed by *Pten*^thyr−/−^ and [*Pten, p53*]^thyr−/−^ mice, respectively.

As predicted by the inability of thyroid-specific *p53* deletion to yield an overt phenotype, a heat map including all probes with more than a 5-fold change across any of the six groups showed that *p53*^−/−^ thyroids cluster together with those of wild type mice (Figure 6A). Similarly, no remarkable differences were apparent between the transcriptomes of *Pten*^thyr−/−^ and [*Pten, p53*]^thyr−/−^ thyroids. On the contrary, the profile of [*Pten, p53*]^thyr−/−^ ATCs (8-10 months of age) was strikingly different from that of younger [*Pten, p53*]^thyr−/−^ mice and also from that of well-differentiated follicular carcinomas developed by aging *Pten*^thyr−/−^ mice (16-20 months). These data strongly suggest that the molecular events leading to the development and maintenance of ATC are unique to this tumor type and that characterization of these changes could uncover clinically relevant pathways and targets.

**Figure 6:** Expression profiling validates the [*Pten, p53*]^thyr−/−^ mouse as a clinically relevant model of human ATC (A) Hierarchical clustering showing the unique expression profile of mouse ATCs when compared to controls, single mutants, ATC-free double mutants (DM), and follicular carcinomas developing in aging *Pten*^thyr−/−^ mice (FTC). (B) Venn's diagram showing the significant overlap between genes differentially regulated in mouse and human ATCs. (C) GSEA analysis of the 430 genes common to mouse and human ATC, showing significant enrichment in genes previously shown to be altered in human ATC cell lines as well as genes involved in the control of mitosis.

Overall, using a stringent false discovery rate (FDR) of 5%, 2,960 genes were found deregulated ±2-fold in ATC samples, compared to wild type thyroids (1,395 up, and 1,565 down). To identify biological processes significantly impacted by ATC development, we performed canonical pathway enrichment using Ingenuity Pathway Analysis (IPA). Significant enrichment was observed in pathways involved in metabolic remodeling of the tumors, in cell motility and invasiveness, in leukocyte recruitment and function, and in epithelial-mesenchymal transition (Table 1).

**Table 1:** Top 25 deregulated pathways identified in mouse ATCs, using the Ingenuity Pathways Analysis (IPA) system

Ingenuity Canonical Pathways	P-value	Ratio	Molecules in pathway
**Hepatic Fibrosis / Hepatic Stellate Cell Activation**	0.00000	0.347	51/147
**Leukocyte Extravasation Signaling**	0.00000	0.276	55/199
**LPS/IL-1 Mediated Inhibition of RXR Function**	0.00000	0.247	54/219
**Propanoate Metabolism**	0.00000	0.190	23/121
**Role of Osteoblasts, Osteoclasts and Chondrocytes in Rheumatoid Arthritis**	0.00000	0.246	59/240
**LXR/RXR Activation**	0.00002	0.280	26/93
**Valine, Leucine and Isoleucine Degradation**	0.00002	0.226	24/106
**Metabolism of Xenobiotics by Cytochrome P450**	0.00003	0.142	28/197
**Atherosclerosis Signaling**	0.00003	0.271	29/107
**Aryl Hydrocarbon Receptor Signaling**	0.00004	0.239	38/157
**Urea Cycle and Metabolism of Amino Groups**	0.00005	0.179	14/78
**Fatty Acid Metabolism**	0.00006	0.179	33/184
**Arginine and Proline Metabolism**	0.00006	0.136	24/177
**Pancreatic Adenocarcinoma Signaling**	0.00006	0.269	32/119
**ILK Signaling**	0.00007	0.238	46/193
**β-alanine Metabolism**	0.00012	0.194	18/93
**Glioma Invasiveness Signaling**	0.00012	0.333	20/60
**Colorectal Cancer Metastasis Signaling**	0.00019	0.218	56/257
**Inhibition of Angiogenesis by TSP1**	0.00019	0.359	14/39
**Cell Cycle Control of Chromosomal Replication**	0.00021	0.387	12/31
**Bladder Cancer Signaling**	0.00022	0.283	26/92
**HIF1α Signaling**	0.00024	0.269	29/108
**Fcγ Receptor-mediated Phagocytosis in Macrophages and Monocytes**	0.00025	0.265	27/102
**IL-8 Signaling**	0.00026	0.223	43/193
**TR/RXR Activation**	0.00068	0.260	25/96

In order to determine to what extent the gene expression changes uncovered in [*Pten, p53*]^thyr−/−^ ATCs overlap with those identified in human anaplastic carcinomas, we retrieved from the GEO and EBI repositories two datasets containing gene expression data from a total of six control thyroids and eight ATCs. Since these two available datasets had been generated using two different Affymetrix platforms [24, 25], we analyzed them separately. After adjusting for a false discovery rate <10% and for genes present in all three platforms, we identified 430 genes that were simultaneously deregulated in all three datasets (Figure 6B and Table 2). An additional 1321 genes were co-deregulated in mouse ATCs and in at least one human dataset.

**Table 2:** Top 50 genes deregulated (FDR<0.1) in both mouse and human ATC, ranked by expression level in mouse

MouseGene	Hs1 ATC	Hs2 ATC	Mm ATC	MouseGene	Hs1 ATC	Hs2 ATC	Mm ATC
	Upregulated				Downregulated		
*Timp1	4.699	5.213	21.086	Patz1	0.436	0.216	0.293
*Steap1	3.760	14.778	10.021	Suox	0.729	0.297	0.291
*Itga5	2.426	4.675	8.795	Epb4.1l4b	0.107	0.029	0.286
**Kif20a**	2.221	22.184	7.664	Tnxb	0.581	0.264	0.285
**Ccnb1**	5.664	11.688	7.395	Fxyd1	0.651	0.307	0.279
Ccna2	3.119	14.546	7.167	Grb14	0.748	0.342	0.276
*Racgap1	7.247	15.876	6.938	1190002H23Rik	0.252	0.212	0.274
Rrm2	10.807	51.614	6.860	Slc5a3	0.220	0.153	0.273
*Prc1	5.295	26.946	6.491	Wwc1	0.384	0.297	0.260
*Tpx2	3.766	38.703	6.390	Mettl7a1	0.090	0.050	0.257
**Kif4**	3.613	19.001	5.861	Stxbp6	0.373	0.044	0.254
**Cenpe**	2.001	13.520	5.749	Tppp	0.681	0.102	0.251
**Cep55**	4.075	26.077	5.707	Acacb	0.527	0.069	0.242
**Kif2c**	2.029	9.175	5.374	Bspry	0.364	0.050	0.237
Ccdc109b	3.470	8.822	5.369	Rbpms	0.370	0.102	0.232
Plau	5.606	46.647	5.363	Cds1	0.516	0.057	0.217
Depdc1a	1.771	7.384	5.303	Nebl	0.112	0.019	0.210
**Bub1b**	3.180	20.421	5.246	Car4	0.273	0.053	0.203
Basp1	3.274	8.466	5.114	*Nkx2-1	0.147	0.016	0.200
Asf1b	1.904	4.015	4.831	Pdk2	0.646	0.474	0.188
Dtl	3.446	5.716	4.782	Bex1	0.178	0.025	0.182
Tyrobp	4.242	19.675	4.652	Sorbs2	0.094	0.013	0.181
**Cdca8**	1.837	6.322	4.577	Cldn3	0.125	0.027	0.180
Rcn1	3.697	2.780	4.547	Sall1	0.287	0.018	0.180
**Cenpa**	1.714	3.183	4.503	Prkcq	0.432	0.134	0.180
**Foxm1**	3.121	7.703	4.434	*Duox2	0.107	0.015	0.178
Nusap1	3.727	17.416	4.385	Rragd	0.222	0.163	0.174
**Dlgap5**	2.449	22.229	4.359	Smad9	0.691	0.024	0.173
Gpsm2	2.351	2.026	4.339	Fabp4	0.102	0.020	0.168
C3ar1	2.891	15.589	4.170	Pygm	0.733	0.605	0.164
**Kntc1**	1.534	7.468	4.146	Gpr56	0.166	0.092	0.161
**Stil**	1.787	6.955	4.098	Rap1gap	0.143	0.028	0.157
**Ncaph**	1.652	4.310	4.088	Erbb4	0.583	0.157	0.150
**Zwilch**	2.346	6.767	4.050	Bex4	0.323	0.148	0.149
Atad2	1.928	2.755	4.000	Glb1l2	0.462	0.270	0.148
Fabp5	7.508	4.293	3.954	Ager	0.683	0.392	0.144
**Cks2**	9.287	26.933	3.911	Lrp2	0.276	0.012	0.133
Tubb6	4.194	4.191	3.839	Ocln	0.650	0.174	0.124
**Cdc20**	5.251	35.621	3.822	Myo5c	0.181	0.046	0.112
Melk	5.470	15.689	3.765	Bcam	0.389	0.246	0.107
**Ttk**	3.254	22.640	3.702	Fam13a	0.304	0.124	0.094
**Aurkb**	1.639	2.222	3.661	Id4	0.050	0.009	0.091
Csf2rb	2.201	22.256	3.632	Fam189a2	0.170	0.015	0.083
Cdkn3	4.688	16.665	3.625	Cdh16	0.305	0.058	0.077
Ube2c	4.383	46.951	3.621	*Ppargc1a	0.362	0.055	0.069
Fcgr2b	2.191	15.069	3.561	*Pax8	0.095	0.014	0.063
Trip13	2.555	14.673	3.418	*Tg	0.011	0.001	0.061
**Ncapg2**	2.384	7.484	3.407	Kcnj16	0.034	0.003	0.045
**Mad2l1**	5.281	15.378	3.398	*Tshr	0.029	0.005	0.045
Mcm3	1.584	2.853	3.366	*Tpo	0.039	0.003	0.036

Strikingly, 24 of the top 50 common up-regulated genes encode for proteins involved in the control of the G2/M transition and of the mitotic process (Table 2, bold), indicating that mitotic deregulation is a key process in the development of ATC, and thus identifying putative clinically valuable targets. As expected, the list of common down-regulated genes contains several thyroid differentiation markers (Table 2, underlined), underlining the dramatic loss of differentiation that characterizes the development of anaplastic thyroid tumors.

To further investigate the 430-gene ATC signature identified by the interspecies analysis, we used Gene Set Enrichment Analysis (GSEA) to query the Molecular Signatures Database (MSigDB), a large collection of curated gene sets [26]. One hundred-nineteen gene sets were enriched in both mouse and human ATCs with an FDR of less than 10%. This included sets of genes up- and down-regulated in anaplastic thyroid carcinoma compared to normal thyroid tissue [27] as well as three independent sets for mitosis-related genes (Figure 6C).

We next used real time PCR to validate a subset of the deregulated genes (marked with an asterisk in Table 2) using an independent set of tissues from control, single mutant, and progressively older double mutant mice, and histology-confirmed ATCs. Dramatic over-expression of the top three genes (ranked based on expression levels in mouse samples), i.e. *Timp1*, *Steap1*, and *Itga5*, was confirmed in mouse ATCs compared to wild type controls, single mutants, and aging double mutants (Figure 7). The expression of *Timp1*, an inhibitor of matrix metalloproteinases that promotes mitogenesis and angiogenesis, and previously found up-regulated in thyroid cancer [28] and of *Steap1*, a cell surface protein found over-expressed in various cancers [29] was already increased (although at a lower level) in *Pten*^thyr−/−^ mice, suggesting a direct role of PI3K signaling in their regulation. Conversely, *Itga5* expression was increased only in ATCs, indicating that integrin α5 may play an active role in the establishment and maintenance of epithelial-to-mesenchymal transition [30]. We also validated the over-expression of *Racgap1*, *Prc1*, and *Tpx2*, which belong to the large group of genes involved in the control of mitosis [31-33]. Validation of the down-regulation of several thyroid differentiation markers is shown in Figure 2. In addition, we validated the striking repression of *Ppargc1a*, the gene encoding for the transcriptional coactivator PGC1-α, which integrates mitochondrial biogenesis and energy production with various cellular functions [34].

**Figure 7:** Real-time PCR validation of a panel of genes differentially regulated in both mouse and human ATCs in 4-month old control and single mutant mice, ATC-free, progressively older (4, 6, 8 months) double mutants, and histologically confirmed ATCs from 8- to 9-month old double mutants

### Mouse ATCs exhibit a glycolytic switch

Many tumors are characterized by a shift from an oxidative to a glycolytic bioenergetic pathway, a phenomenon known as the Warburg effect [35]. Human ATCs commonly display intense glucose uptake on ^18^F-FDG PET imaging, indicating that this tumor type has a strong glycolytic phenotype [36].

The down-regulation of *Ppargc1a* prompted us to test whether the ATCs developing in [*Pten, p53*]^thyr−/−^ mice reflect this metabolic shift. We performed ^18^F-FDG PET imaging on sex- and age-matched control and ATC-bearing mice (8-month old), and found that tumor-bearing [*Pten, p53*]^thyr−/−^ mice avidly uptake radiolabeled glucose (Figure 8A). Furthermore, immunohistochemical, western blotting, and real time PCR approaches revealed that ATCs developing in [*Pten, p53*]^thyr−/−^ mice consistently up-regulate *Hif1α*, *Hexokinase 2*, and *Pyruvate Kinase M2*, all of which have been shown to be directly responsible for the establishment of the Warburg effect (Figure 8B-D). Although *Ldha*, the gene encoding Lactate Dehydrogenase A, was not consistently up-regulated in mouse ATCs, we found that lactate content of every tumor tested was dramatically increased (up to four-fold) compared to control thyroids, further demonstrating the highly glycolytic nature of these tumors (Figure 8E).

**Figure 8:** Mouse ATCs undergo a glycolytic switch (Warburg effect) (A) Coronal section (transverse in the inset) of representative ^18^FDG PET scans of 8-month old control and compound mutant mice, showing high ^18^FDG accumulation in the thyroid tumor. (B) H&E and immunohistochemical detection of Hexokinase II and Pyruvate kinase M2 in the anaplastic component of a representative mouse tumor. The line demarcates the boundary between well-differentiated and anaplastic component. (C) Western blotting showing the increased expression of Hif1α, Hexokinase II and Pyruvate kinase M2 in four mouse ATCs (T1-T4). (D) Real-time PCR analysis of the expression of Hexokinase II, Pyruvate kinase M2, and Lactate dehydrogenase A in five mouse ATCs (T1-T5). (E) Lactate content of four wild type thyroids and five ATCs (T1-T5), showing consistent increase in neoplastic glands.

### Mouse and human ATC cell lines are sensitive to glycolytic inhibitors

Based on these results, we tested whether the glycolytic inhibitor 2-deoxyglucose (2-DG), a glucose analogue which is phosphorylated by hexokinase but cannot be further metabolized in the glycolytic process [37], would affect the growth and survival of two cell lines we established from ATCs developed by [*Pten, p53*]^thyr−/−^ mice. Both cell lines were efficiently inhibited by 2-DG, showing dose-dependent growth suppression at 48h with an ED_50_ (0.3 mM for T1860 and 1.8 mM for T1903) remarkably lower than previously reported (6.7-8.1 mM) for prostate and breast cancer cell lines [37] (Figure 9A, top panels), suggesting that ATC cells might be especially sensitive to glycolysis inhibition. However, glycolytic inhibitors as single agents have shown limited efficacy *in vivo* [38], while their combination with standard chemotherapy has shown, in some instances, a promising synergistic effect [38, 39]. Thus we tested whether 2-DG could enhance the cytotoxic effect of doxorubicin, a standard, although poorly effective, treatment for ATC. We compared the single agent dose-response curves of the two aforementioned mouse ATC cell lines to the curve obtained using the two drugs combined at a fixed ratio based on the most effective single dose concentration for each drug. The combination treatment was more effective than each single agent over a wide range of concentrations (Figure 9A, middle panels). In order to establish whether the combined effects of 2-DG and doxorubicin were synergistic rather than additive, we calculated the combination index (CI) according to the well-established Chou and Talalay median effect method [40]. Figure 9A (bottom panel) shows the isobolograms for the drug combinations in the two cell lines, and the calculated CIs for the ED_50_. Strong synergistic effects (CI<1) resulted from the combination of 2-DG and doxorubicin.

**Figure 9:** Both mouse and human ATC cell lines are highly sensitive to glycolytic inhibitors (A) Top panel: dose-response curves showing the effect of 2-deoxyglucose (2-DG) on the viability of two mouse ATC cell lines. Middle panel: dose-response curves showing the. Bottom panel: isobolograms showing strong synergy between the two compounds. (B) Top panel: dose-response curves showing the cooperative effect of a 2-DG/Doxorubicin combination on the viability of two human ATC cell lines. Middle panel: isobolograms showing strong synergy between the two compounds. (C) Isobolograms showing strong synergy between doxorubicin and another glycolytic inhibitor, 3-bromopyruvate (3-BP).

Next, we extended these findings to two human ATC cell lines, CAL-62 and C643, characterized by different *driver* mutations compared with our mouse model. CAL-62 harbors a G12R *KRAS* mutation, while C643 harbors a G13R *HRAS* mutation [41]. In addition, p53 is inactivated in both cell lines, consistent with most ATCs [42].

Both human ATC cell lines responded to 2-DG in a manner similar to the mouse cells, with an ED_50_ (0.48 mM for CAL-62, 1.19 mM for C643) again lower than previously reported for other tumor types (Figure 9B, top panels). Doxorubicin alone was more effective in CAL-62 than in C643. When combined in a fixed ratio, the two drugs displayed a striking increase in efficacy at all concentrations tested, and the CI calculation confirmed the strongly synergic nature of this interaction (Figure 9B, bottom panels).

To conclusively demonstrate that inhibition of glycolysis can effectively synergize with standard chemotherapy in ATC, we used a second glycolysis inhibitor, 3-bromopyruvate (3-BP), an alkylating agent that inhibits hexokinase and GAPDH [43]. Since 3-BP has a Ki for glycolysis inhibition of 2.4 mM, while the one for DG is 15.5 mM, 3-BP appears to be a more efficient glycolysis inhibitor than 2-DG [44]. When combined with doxorubicin, 3-BP showed a strong synergistic effect, with a CI of 0.3 (Figure 9C).

Taken together, these data strongly suggest that anaplastic thyroid carcinomas are highly sensitive to glycolysis inhibitors, especially in combination with cytotoxic chemotherapy, independent of the nature of the driver mutation originally responsible for the transformation process.

## DISCUSSION

The prevalence of thyroid cancer is increasing worldwide, and this is due only in part to improved and earlier detection [45]. Although less than 5% of the 48,020 new thyroid cancer cases (+7.5% compared to 2010) estimated for 2011 in the United States [46] will be diagnosed as anaplastic tumors, the latters will account for the majority of the 1,740 estimated annual deaths. The dismal prognosis associated with these tumors reflects their intrinsic resistance to any therapeutic approach, including surgery, radiation, chemotherapy, and targeted therapy [6]. The genomic instability and karyotypic complexity that characterize ATCs [12] are likely major determinants of therapy resistance, since they result in the simultaneous activation of multiple oncogenic pathways, and thus in the establishment of a redundant network offering multiple escape and survival routes. All our current knowledge on the pathogenetic mechanisms of ATC is based on the analysis of patient material and on the use of cell lines and xenograft models. It is thus clear that an *in vivo*, immunocompetent, and clinically relevant model of ATC would be a critical tool to better understand the mechanisms associated with ATC development, and to identify novel, more effective therapeutic targets.

Most ATCs harbor mutations that activate one of two pathways that act as *drivers* of the transformation process: the RAS/BRAF/MAPK cascade, and the PI3K/PTEN/AKT cascade [47]. These mutations are usually already present in the well-differentiated tumor component from which most ATCs develop [3, 4]. In addition, most ATCs share inactivating mutations of *p53*, which are likely to determine, in combination with the driver mutations, the anaplastic features of these tumors [48].

Building upon these patient-derived genetic data, we have generated the first mouse model of ATC by combining, in the mouse thyroid follicular cells, *p53* loss with constitutive PI3K activation, via deletion of the *Pten* tumor suppressor.

The most clinically relevant feature of this model is the remarkable similarity of its morphological and molecular features to human ATCs, including those tumors that do not display PI3K activation. [*Pten, p53*]^thyr−/−^ anaplastic tumors derive from pre-existing follicular carcinomas, and exhibit cellular pleomorphism, aneuploidy, genomic instability, and epithelial-to-mesenchymal transition. This latter feature is of particular interest, since recent data in the breast and other tissues suggest that EMT is linked to the generation of a cancer-initiating cell (or cancer stem cell) population [49, 50], endowed with an intrinsic drug resistance phenotype [51]. Ongoing studies in this model will shed more light on the signals and mechanisms that initiate and maintain this phenotype.

The expression of all the classical thyroid-specific markers, including that of the sodium-iodide symporter (NIS), is lost as a consequence of the de-differentiation process. Thus this model provides us with a novel *in vivo* tool to explore the mechanisms leading to NIS suppression, and to attempt to pharmacologically restore radioiodine sensitivity, as recently described in a model of papillary and poorly differentiated *BRAF*^V600E^-dependent thyroid carcinoma [52].

Another important and clinically relevant feature of our model, underlining its high similarity to human tumors, is the absence of the dramatic TSH increase typical of all current mouse models of advanced thyroid cancer, a phenotype that is never seen in human patients [15, 18, 52]. The possible confounding effects of high TSH levels during the transformation process are underlined by the absence of neoplastic transformation when these models are crossed to *Tshr*^−/−^ mice [17, 53].

Despite the simultaneous loss of *Pten* and *p53*, it still takes at least 6 months for these mice to develop frank carcinomas, which might suggest the need for additional genetic alterations to accumulate. Our data exclude the presence of mutations in the hotspots of known ATC-related genes (*Braf*, *H-*, *N-*, and *Kras*), and indicate that a thorough, genome-wide approach to identify possible additional cooperating events is warranted.

A noteworthy feature, with important clinical implications, is that although ATCs are aneuploid and genomically instable, and thus resistant to single agent approaches, still they are somewhat addicted to their original driver mutation. In fact, a well characterized AKT inhibitor, MK-2206, was much more effective on cell lines derived from murine [*Pten, p53*]^thyr−/−^ anaplastic tumors than on human cell lines harboring *RAS* mutations. Although this notion will need additional in-depth validation, it might represent a valid rationale for the use of driver pathway-targeted inhibitors in combination with cytotoxic drugs.

Further support to the clinical relevance of this model comes from the analysis of its molecular features. Expression profiling of control, single, and double mutant thyroid glands, compared with follicular and anaplastic tumors developed by *Pten*^thyr−/−^ and [*Pten, p53*]^thyr−/−^ mice respectively, revealed a substantial similarity between *Pten*^thyr−/−^ and [*Pten, p53*]^thyr−/−^ hyperplasias and *Pten*^thyr−/−^ follicular carcinomas, emphasizing the driver role of PI3K activation in the establishment of neoplastic transformation. Strikingly, ATC profiles were significantly different from any other sample, including younger [*Pten, p53*]^thyr−/−^ compound mutants, underlining the existence of a dramatic biological switch associated with the establishment of anaplasia and EMT. Molecular characterization of this switch will undoubtedly yield much-needed clues on potential therapeutic targets along the pathways involved. While the biological features of ATCs predicted an enrichment in genes involved in pathways related to EMT, invasion, and metastasis, it is interesting that we also found significant alterations in groups of genes associated with metabolic pathways, such as *Propanoate metabolism*, *Urea cycle*, and *Arginine and proline metabolism*, that have been recently associated with a neoplastic state [54].

Analysis of the overlap between genes significantly deregulated in our mouse model and those deregulated in the only two Affymetrix-based, publicly available, datasets containing human ATCs [24, 25] has allowed us to define a set of 430 genes consistently and significantly deregulated in both mouse and human ATCs. Strikingly, this “ATC signature” is highly enriched in genes encoding proteins involved in the control of mitosis, and shows a considerable overlap with the “cell proliferation and chromosomal instability signature” reported by Salvatore *et al.* using a different platform [12]. The availability of novel, specific inhibitors of key mitotic kinases such as Aurora A [55] and Plk1 [56] emphasizes the clinical relevance of this finding, and, together with preliminary reports showing efficacy of Plk1 inhibition in ATC cell lines [57], warrants further studies in ATC models using these compounds alone or, more likely, in combination with other relevant drugs.

Finally, we have provided evidence that, similar to human ATCs, [*Pten, p53*]^thyr−/−^ tumors are highly glycolytic and very sensitive to two compounds, 2-DG and 3-BP, targeting different steps of glycolysis. Despite a growing literature supporting the efficacy of anti-glycolytic compounds in cancer cell lines [37, 39, 58] as well as in xenograft models [38, 44], their clinical development as single agents has been slowed down by toxicity-related issues associated with prolonged administration of high concentrations of these drugs. However, promising results have been obtained in clinical trials using 2-DG as a radiosensitizer [59]. More specific inhibitors, with the goal of widening their therapeutic window, are currently under development [60]. Our data support the notion that glycolysis inhibitors not only decrease proliferation and survival of ATC cells as single agents at a relatively low concentration, but also significantly increase the efficacy of a cytotoxic drug, doxorubicin, already in clinical use for ATC. The rationale for this combination is twofold: i) DNA damage caused by doxorubicin cannot be effectively repaired when the cell's ATP levels are reduced upon glycolytic inhibition; ii) reduced ATP will decrease the efficacy of the ATP-dependent pumps responsible for the efflux of doxorubicin from the cells. Thus, our proof-of-principle data provide a strong rationale to develop and test additional combinations of novel glycolytic inhibitors and clinically relevant chemotherapeutic drugs in sensitive tumor types, such as ATC, for which current therapeutic approaches invariably fail.

## METHODS

### Animals

The *Pten^L/L^* and TPO-Cre strains have been described [22]. All strains were backcrossed in the 129Sv background for at least eight generations, and littermates were used as controls.

### Hormone measurements

Blood was collected by cardiac puncture. Serum thyroid-stimulating hormone (TSH) was measured using a sensitive, heterologous, disequilibrium double-antibody precipitation RIA [61], and results were expressed in mU/liter. All samples were individually analyzed for each mouse. Total T4 concentrations were measured by a solid-phase RIA (Coat-a-Count; Diagnostic Products Corp., Los Angeles, CA) adapted for mice. Values of the respective limits of assays sensitivities were assigned to samples with undetectable TSH and T4 concentration.

### Immunohistochemistry

6 μm sections were subjected to antigen retrieval, incubated with pERK1/2 (Thr202/Tyr204), pAKT (Ser473), pSmad2 (Ser465/467), Vimentin, e-Cadherin, HK2, and PKM2 antibodies (Cell Signaling, Danvers, MA) and counterstained with hematoxylin.

### Establishment and maintenance of cell lines

Primary thyroid tumors were minced and resuspended in Ham's F12/10% FBS with 100 U/ml type I collagenase (Sigma, St. Louis, MO) and 1 U/ml dispase (Roche, Indianapolis, IN). Enzymatic digestion was carried out for 90 min at 37°C. After digestion, cells were seeded in Ham's F12 containing 40% Nu-Serum IV (Collaborative Biomedical, Bedford, MA), gly-his-lys (10ng/ml, Sigma), and somatostatin (10ng/ml, Sigma) and allowed to spread and reach confluence before being passaged. After the fourth passage, tumor cells were adapted to grow in DMEM/10%FBS.

### Mutation detection

Genomic DNA was isolated from cell lines established from primary tumors and subjected to PCR to amplify fragments suitable for sequencing [62]. PCR products were gel purified and sequenced from both ends.

### Metaphase preparation and chromosome analysis

For chromosome preparation, primary cells at passage p1-p3 were plated in a 35mm Petri dish and incubated with Colcemid (Sigma Aldrich, St. Louis, MO) at a concentration of 10 ng/ml over night or for 3hrs at 100 ng/ml. Chromosomes were extracted with standard hypotonic treatment (0.075 M KCl), dropped on microscope slides and mounted with antifade containing DAPI (Invitrogen, Carlsbad, CA). Slides were imaged on a Zeiss Axiovert 200 Microscope using a DAPI filter (Chroma Technologies, Bellows Falls, VT). Ten fields were selected randomly and 15 to 30 cells for each tumor line were subjected to chromosome count and visually inspected for the presence of gross chromosome abnormalities and chromosome fragments.

### Western blot analysis

Thyroids and cells were homogenized on ice in RIPA buffer supplemented with Complete protease inhibitor tablet (Roche Diagnostics, Indianapolis, IN). Western blot analysis was carried out on 20-40 μg proteins using phospho-antibodies from Cell Signaling (Danvers, MA) and a β-actin antibody from Sigma-Aldrich.

### Drug treatments

Pharmacological inhibitors of AKT (MK-2206, Selleck Chemicals), and MEK1/2 (U0126, Cell Signaling) were added 24h after plating, in sextuplicate. After 72h, viability was assessed using the Wst-1 assay (Takara) and IC50s were determined using Prism software.

### Real time PCR

Total RNA was extracted with Trizol and reverse transcribed using the Thermoscript kit (Invitrogen). qRT-PCR was performed on a StepOne Plus apparatus using the Absolute Blue qPCR Rox Mix (Thermo Scientific, Waltham, MA) and TaqMan expression assays (Applied Biosystems, Carlsbad, CA). Each sample was run in triplicate and *Ipo8* was used to control for input RNA. Data analysis was based on the Ct method, and experiments were repeated at least three times using at least two independent organ pools (at least five mice/pool).

### Expression profiling

Three pools of three to five mice, and five individual, flash-frozen, histologically verified tumor samples of each histotype, were randomly selected from each of the six different groups (control, *Pten*^thyr−/−^, *p53*^thyr−/−^, [*Pten, p53*]^thyr−/−^, follicular carcinomas, anaplastic carcinomas). Tumor fragments and thyroid glands were subjected to total RNA isolation using TRIzol Reagent (Invitrogen) followed by further purification with the RNAeasy Kit (Qiagen). Total RNA quality was verified using the Agilent Bioanalyzer 2100. Microarray hybridization was performed at the Albert Einstein Genomics Facility using Affymetrix Mouse Gene 1.0 arrays. Normalization and background subtraction were performed with RMA, using the “oligo” package of Bioconductor. Gene selection was performed using the “limma” package. Raw p values were corrected for multiple testing using a “false discovery rate” < 0.05. Microarray data were deposited in GEO (accession no. GSE30427).

### Canonical Pathway Analysis

Canonical pathways analysis identified the pathways from the Ingenuity Pathways Analysis library of canonical pathways that were most significant to the data set. Molecules from the data set that met the ±2-fold cutoff with a FDR<0.05 and were associated with a canonical pathway in Ingenuity's Knowledge Base were considered for the analysis. The significance of the association between the data set and the canonical pathway was measured in 2 ways: 1) A ratio of the number of molecules from the data set that map to the pathway divided by the total number of molecules that map to the canonical pathway. 2) Fisher's exact test was used to calculate a p-value determining the probability that the association between the genes in the dataset and the canonical pathway is explained by chance alone.

### Interspecies analysis

Two human datasets were obtained from GEO (E-GEOD-27155: 4 normal vs. 4 ATC) and EBI (E-MEXP-2442: 2 normal vs. 4 ATC). The mouse dataset (see above) contained six independent wild type pools and 5 individual ATCs. .CEL files were processed and normalized using the RMA function and the “affy” and “oligo” packages of Bioconductor. Data for each experiment were normalized separately, due to the different Affymetrix platforms used in the three experiments. Gene selection for each experiment was done using the “limma” package. Raw p values were corrected for multiple testing using a “false discovery rate” <0.1. Top tables were generated for all probe-sets for each experiment. Human-mouse homology mapping file were obtained from the MGI database (ftp.informatics.jax.org/pub/reports/HMD HGNC Accession.rpt) and 11,508 genes common to all three datasets were selected.

### Lactate assay

Lactate levels were assayed using a commercially available kit (Biovision, Mountain View, CA). Lactate levels were normalized to the amount of DNA extracted from each tissue fragment.

### [^18^F]Fluorodeoxyglucose positron emission tomography imaging

Wild type and [*Pten*, *p53*]^thyr−/−^ mice were fasted overnight before a tail vein injection of [^18^F]fluorodeoxyglucose (300 μCi). One hour after injection, mice were subjected to positron emission tomography (PET) scanning with the Concorde Microsystems R4 microPET Scanner. Animals were imaged while anesthetized through inhalation with isoflurane. Image acquisition was done using the MicroPET Manager with the ASPIRO dedicated software.

### Chemotherapic treatments

Doxorubicin (Sigma) and glycolytic inhibitors, 3-Bromopyruvate and 2-Deoxyglucose (Sigma) were added 24h after plating, in quadruplicate. After 48hs cell viability was assessed using the Wst-1 assay (Roche). Preliminary experiments were conducted to ensure that, in the conditions used for these assays, this method yields the same results as direct cell counting (both trypan blue-based and automated).

### Analysis of synergy

Doxorubicin was combined with each of the different glycolytic inhibitors at a fixed ratio (1:1) of the individual IC90 concentrations of each drug. Drug combinations were then serially diluted. Statistical analysis of drug synergy was evaluated from the results of the Wst-1 assays and calculated using the Chou-Talaly method [40] and the Calcusyn Software (Biosoft). To determine synergy between two drugs, the software uses a median-effect method that determines if the drug combination produces greater effects together than expected from the summation of their individual effects. The combination index (CI) values are calculated for the different dose-effect plots (for each of the serial dilutions) based on the parameters derived from the median-effect plots of the individual drugs or drug combinations at the fixed ratios. The CI was calculated based on the assumption of mutually nonexclusive drug interactions. CI values significantly > 1 are antagonistic, not significantly different than 1 are additive, and values < 1 are synergistic.

### Statistical analysis

Experiments were performed at least three times. Data were analyzed using the JMP 5.1, Calcusyn, and Prism software packages. Differences with P-values <0.05 were considered statistically significant.
